# Assessing the Readability of Anesthesia-Related Patient Education Materials from Major Anesthesiology Organizations

**DOI:** 10.1155/2022/3284199

**Published:** 2022-07-13

**Authors:** Anna Pashkova, Raksha Bangalore, Cynthia Tan, Peter F. Svider, Anna Korban, Yee-Kuen Yam, Faraz Chaudhry, Jean Anderson Eloy, Jean Daniel Eloy

**Affiliations:** ^1^Department of Anesthesiology, Rutgers University, New Jersey Medical School, Newark, New Jersey, USA; ^2^Department of Otolaryngology-Head & Neck Surgery, Rutgers University, New Jersey Medical School, Newark, New Jersey, USA; ^3^Department of Neurological Surgery, Rutgers University, New Jersey Medical School, Newark, New Jersey, USA; ^4^Center for Skull Base and Pituitary Surgery, Rutgers University, New Jersey Medical School, Newark, New Jersey, USA

## Abstract

**Introduction:**

The National Institutes of Health (NIH), American Medical Association (AMA), and the US Department of Health and Human Services (USDHHS) recommend that patient education materials (PEMs) be written between the 4th to 6th grade reading level to ensure readability by the average American. In this study, we examine the reading levels of online patient education materials from major anesthesiology organizations.

**Methods:**

Readability analysis of PEMs found on the websites of anesthesiology organizations was performed using the Flesch Reading Ease score, Flesch-Kincaid Grade Level, Simple Measure of Gobbledygook, Gunning Frequency of Gobbledygook, New Dale-Chall test, Coleman-Liau Index, New Fog Count, Raygor Readability Estimate, the FORCAST test, and the Fry Score.

**Results:**

Most patient educational materials from the websites of the anesthesiology organizations evaluated were written at or above the 10th grade reading level.

**Conclusions:**

Online patient education materials from the major anesthesiology societies are written at levels higher than an average American adult reading skill level and higher than recommended by National Institute of Health, American Medical Association, and US Department of Health and Human Services. Online resources should be revised to improve readability. Simplifying text, using shorter sentences and terms are strategies online resources can implement to improve readability. Future studies should incorporate comprehensibility, user-friendliness, and linguistic ease to further understand the implications on overall healthcare.

## 1. Introduction

The American Society of Anesthesiologist (ASA) estimates 40 million anesthetics are administered yearly in the United States. Although patients have greater preoperative access to their surgeons, many do not meet their anesthesiologists until the day of their procedure, placing special importance on the availability of appropriate resources specific to any questions and concerns they have regarding risks, complications, and other anesthesia-specific topics. Patient educational materials (PEMs) have become ubiquitous with the popularization of the Internet as a health information resource. Nearly 8 out of 10 adults in the United States report looking up information on the Internet about health topics [1].

Americans use the Internet as a tool to better inform themselves about diseases and conditions in all of the medical specialties and as such designing online-based PEMs so they can be reliably interpreted by the average layperson has become of ultimate importance [2]. The average American adult reads between an estimated 6th to 8th grade level [3–6]. In light of these literacy levels, the National Institutes of Health (NIH), American Medical Association (AMA), and US Department of Health and Human Services (USDHHS) have published recommendations outlining that PEMs should be written at a 4th to 6th grade reading level [7–9]. Formulating comprehendible PEMs has profound implications on costs and health outcomes. Patients with deficiencies in “health literacy,” defined as the skills essential to function effectively in a healthcare setting, including reading and comprehension, have higher rates of adverse patient outcomes, such as longer hospital stays, additional hospitalizations, and more frequent emergency care visits [10–16].

Readability estimates can be performed using several commonly used assessments [16–18]. To the best of our knowledge, there are no studies assessing readability of online-based anesthesia PEMs. Our objective was to use the readability assessment tools outlined in Methods to evaluate the online PEMs from the ASA, as well as a comparison of these resources to PEMs from other associated societies listed on their website, including the Society of Cardiovascular Anesthesiologists (SCA) and the American Society of Regional Anesthesia and Pain Medicine (ASRA). Additionally, comparison to online PEMs from the Canadian Anesthesiologists' Society (CAS) was performed.

## 2. Methods

Online PEMs were found on the ASA's patient information website, Lifeline to Modern Medicine (http://www.lifelinetomodernmedicine.com/). Once the ASA PEMs were obtained, they were divided into the following general categories, agreed upon by two independent reviewers: background information, critical care anesthesia, geriatric anesthesia, obstetric anesthesia, pain management, pediatric anesthesia, and risks and complications (Table 1). Any grammatical symbols such as semicolons, decimals, bullets, and abbreviations were removed prior to analysis. Readability assessments were conducted using Readability Studio Professional Edition Version 2012.1 for Windows (Oleander Software, Ltd. These instruments are not copyrighted, no permission required for use. Vandalia, OH). Any text that contained nonmedical information, such as citations, references, copyright notices, or advertisements was excluded from this analysis. The readability assessments including Raygor Readability Estimate, FORCAST test, Fry Score, Coleman-Liau Index (CLI), the New Fog Count (NFC), Simple Measure of Gobbledygook (SMOG), Flesh-Kincaid Grade Level (FKGL), Flesch Reading Ease (FRE) score, New Dale-Chall (NDC) test, and the Gunning Frequency of Gobbledygook (G-FOG) were used to estimate grade level and difficulty among the analyzed PEMs. The Raygor Readability Estimate takes into account the average number of sentences and lengthy words to make a visual representation of grade level [19]. The FORCAST test quantifies single-syllable words and calculates a grade level, while the Fry test uses the number of syllables and sentences to illustrate grade level on a graph [20]. The Coleman-Liau score takes into account sentence length and character count, while the New Fog Test considers sentence length and the use of polysyllabic words (words > 4 syllables) [21]. The SMOG test also considers polysyllabic words, along with sentence length, to determine a grade level [22]. The FRE uses syllable count and sentence length to provide a score depicting difficulty between 0 and 100, a score of 0 being the easiest and 100 being most difficult. The FKGL supplements the difficulty with an estimated grade level [23, 24]. The NDC test uses the number of unfamiliar words, meaning those not found on a list of words commonly used and comprehended by 4th graders, along with sentence length [21]. The Gunning-Fog assessment uses polysyllabic words (defined as “complex”) and total number of sentences to determine a grade level based on American standards [22]. As a secondary analysis, the aggregate of the text from the ASA PEMs was pasted into a single Microsoft Word document and compared with PEMs from other organizations listed on the ASA website, including the SCA and ASRA, as well as to web-based PEMs from the CAS. The same software and readability assessments were used for this analysis and cross verified by two individuals. All PEMs obtained, including those from the ASA, SCA, ASRA, and CAS, were accessed in June 2021.

## 3. Results

Grade-level estimates calculated from the readability assessments indicated that difficulty of PEMs from the ASA website averaged at the 11th grade level and above for all topics (Figure 1), although there was variation among the individual readability assessments (Table 2). The FRE readability chart indicated that the PEMs from all topics were at the “difficult” or “very difficult” level (Figure 2). The Raygor Readability Estimate, depicted visually, indicates that all topics were written at or above a 10th grade reading level (Figure 3). The same readability assessments were performed comparing PEMs from the ASA, CAS, SCA, and ASRA. PEMs from the websites of these organizations were written on average above a 12th grade reading level (Figure 4), although variation was exhibited among the individual readability assessments as well (Table 3). The FRE readability chart and the Raygor Readability Estimate are depicted visually in Figures 5 and 6, respectively.

## 4. Discussion

The rapid expansion of the Internet over the past two decades has allowed for unprecedented access to information describing a myriad of medical conditions and treatments. Elderly patients and those in lower socioeconomic classes are most vulnerable to deficits in health literacy and subsequent poorer health outcomes [25–27]. As a result, decisions regarding strategies for designing appropriate PEMs have potentially widespread ramifications. Creating online-based PEMs that are readily understood by the average American adult who reads at a 6th-8th grade level is a reasonable and necessary objective, since currently, both private and governmental health organizations are seeking ways to increase health efficiency. By making online-based PEMs more comprehendible, patients will be better informed about decisions on whether to seek care, including details as specific as warning signs for acute medical emergencies. In anesthesiology, access to appropriately written PEMs can help patients better understand perioperative risks, as well as stress the importance of patient participation in maximizing safety. For example, one systematic review revealed that smoking cessation at least 4 weeks prior to anesthetic administration resulted in a 0.56 risk ratio for postoperative complications [28]. Patient-oriented techniques that take time to implement, such as smoking cessation and weight loss, would be especially useful to convey via PEM, since education on the day of the procedure via the anesthesiologist would be of little use. Patients can also learn more about what type of information about past medical history is important to report to their anesthesiologist preoperatively, decreasing associated risks if this information is not elicited during preoperative assessment.

There are several clear-cut strategies that can be employed by the creators of anesthesia PEMs to simplify the text and better communicate information to patients. These tactics include, but are not limited to, using simpler and shorter words, shorter sentences, and stating health information in fewer total sentences. Readability tests used in this evaluation mostly assessed these same properties of the online PEMs when calculating grade-level difficulty. As an example of this, here is a passage from an ASA PEM that can be improved using these strategies: “Because the risks are different for each patient, there is no single way to manage against anesthesia risk factors. However, we encourage you to work with your medical team – including your physician and anesthesiologist – before any procedure takes place. For example, if you are a smoker and you are scheduled for surgery, anesthesiologists recommend that you take steps right away to quit and remain smoke-free until at least one week after your procedure. Smokers have a greater chance of developing complications, including wound infections, pneumonia and heart attacks, both during and after surgery. The sooner you quit smoking before surgery, the better your chances are of avoiding complications.”

This passage was written at between a 13th and 14th grade reading level, averaging the scores of the readability assessments. By simplifying and shortening this passage to the following, the difficulty was decreased to a 6th grade reading level: “Each patient is unique. Talk to all your doctors before the procedure. Quit smoking at least one week before the procedure. Smoking is a risk for wound and lung infections, and heart attacks. These can happen during or after the procedure. The sooner you quit smoking, the less risk there is.”

This edited passage meets the guidelines from the NIH, AMA, and USDHHS recommending all PEMs be written at between the 4th and 6th grade reading levels. Articles from the ASA website were, on average, far more difficult than the reading grade level, along with data from the FRE score. There was some variability upon examining data from the individual readability assessments, with the vast majority of them still indicating challenging grade reading levels. Upon comparison of the average readability level of ASA documents to PEMs from other organizations, the ASA PEMs were written at equivalent or slightly easier levels, with the CAS and SCA's documents having the highest grade-level readability figures. The findings from this study allow for the comparison between the various anesthesia organizations with readily available online PEMs, along with an internal comparison of ASA patient resources. However, the most important point to stress in this analysis is that all of these anesthesia PEMs were written well above the reading level of the average American, and even further above the 4th to 6th grade level recommended by the NIH, AMA, and USDHHS guidelines. Currently available anesthesia PEMs from these popular resources should be simplified not only to allow for greater understanding and reassurance about conditions, but also because of the potential for subsequent improvements in patient outcomes.

Our analysis had a few limitations. Certain formats of PEMs such as videos and pictures were excluded from our study. Online PEMs from only 4 organizations were analyzed. Although these are robust online sources of information and represent some of the most influential societies in anesthesiology, there are many other sources of information that patients can be directed to for this purpose. In addition, readability formulas are limited in assessing for comprehensibility of a written matter and do not take into consideration individual reader factors such as cultural, socioeconomic, and religious which may affect overall understanding. The readability formulas used in our analysis also do not consider if PEMs explain scientific terms for the reader nor the user-friendliness of the PEMs by the reader. Future studies incorporating comprehensibility, user-friendliness, and linguistic ease in addition to readability are indicated to further understand the implications on overall healthcare.

## 5. Conclusion

The findings from these readability assessments suggest that available online PEMs from these major anesthesiology societies, including the ASA, the CAS, the SCA, and the ASRA, are written at a reading level too complicated for the average American. These online resources should be revised and written with improved readability and accessibility for all patients which may lead to more informed decisions and potentially better health outcomes. Future studies should assess readability in combination with comprehensibility and user-friendliness to better understand the implications on how the patient experience of PEMs impacts their overall healthcare.

## Figures and Tables

**Figure 1:** Mean estimated grade level of patient educational materials from the American Society of Anesthesiologists website (https://www.lifelinetomodernmedicine.com).

**Figure 2:** Flesch Readability chart illustrating that most categories of articles analyzed from the American Society of Anesthesiologists' website were in the “difficult” to “very difficult” classification of readability.

**Figure 3:** Raygor Readability Estimate graph illustrating the grade-level difficulty of patient education materials from the American Society of Anesthesiologists' website.

**Figure 4:** Mean estimated grade level of patient educational materials from the American Society of Regional Anesthesia and Pain Medicine, American Society of Anesthesiologists, Canadian Anesthesiologists' Society, and Society of Cardiovascular Anesthesiologists.

**Figure 5:** Flesch Readability chart illustrating that patient education materials analyzed from the websites of the American Society of Regional Anesthesia and Pain Medicine, American Society of Anesthesiologists, Canadian Anesthesiologists' Society, and Society of Cardiovascular Anesthesiologists were in the “difficult” to “very difficult” classification of readability.

**Figure 6:** Raygor Readability Estimate graph illustrating the grade-level difficulty of patient education materials from the websites of the American Society of Regional Anesthesia and Pain Medicine, American Society of Anesthesiologists, Canadian Anesthesiologists' Society, and Society of Cardiovascular Anesthesiologists.

**Table 1:** Articles from the American Society of Anesthesiologists' patient information website, Lifeline to Modern Medicine.

*Background (12)* Know your anesthesia provider before surgery Propofol as anesthesia Facts about anesthesia providers and your safety Say NO Colorado (about CRNAs and supervision) Tips for patients considering ambulatory surgery QA what you should know before surgery Anesthesiology 101: what do I need to know Common questions for patients preparing for anesthesia Herbal and dietary supplement use Medical tourism Medical tourism questions to ask Q&A medical tourism *Critical care anesthesiology (3)* Trauma Medically induced coma vs. sedation Transplant anesthesia	*Risks and complications (18)* Anesthesia and malignant hyperthermia Q&A malignant hyperthermia Anesthesia awareness Ambulatory surgery safety Obesity and anesthesia Obstructive sleep apnea Operating room fires Stop smoking Reaction to anesthesia Facts about malignant hyperthermia Facts about OSA 7 things to know about anesthesia awareness Anesthesia drug shortages and you Anesthesiology and weight-loss surgery Obese patients and ambulatory surgery centers Q&A stop smoking Why and how to quit smoking Understand the risks of anesthesia
*Pediatric (7)* Children and surgery Pediatric obesity and anesthesia Robo tripping and children FAQ: Robo tripping/OTC drug abuse Q&A for parents: your child's surgery Steps for preparing your child for surgery Does anesthesia affect my child?	*Obstetric anesthesia (7)* Labor and delivery Nitrous oxide during labor Q&A: chronic pain Obesity and pain management during childbirth Potential epidural side effects and risks Tips to help ease the discomfort of childbirth Types of pain relief in labor and delivery
*Pain management (5)* Pain medicine Anesthesiologists in pain medicine Q&A cancer pain Q&A acute postoperative pain medicine Treatments for managing pain	*Geriatric anesthesia (4)* Seniors Q&A geriatric anesthesia Alzheimer's disease and anesthesia Surgical checklist for seniors and caregivers

All articles were grouped into the categories (background, critical care anesthesiology, risks and complications, pediatric, obstetric anesthesia, pain management, and geriatric anesthesia) created by the authors. These individual articles do not appear organized by these categories on Lifeline to Modern Medicine. All articles were accessed June 2021.

**Table 2:** Readability assessment scores of patient education materials from the American Society of Anesthesiologists.

Category	CLI	NDC	FKGL	FCS	Fry	G-FOG	NFC	SMOG
Background	14.1	11-12	12.7	11.6	17	14.3	8.9	14.6
Critical care	14.8	13-15	14.9	12.2	17	16.3	13	15.2
Geriatrics	12.4	11-12	11.7	11.1	16	13.5	7.3	14.2
Obstetrics	11.1	9-10	10.9	11	12	11.9	8.3	12.8
Pain Mgmt	13.4	11-12	12.2	11.4	15	12.4	7.8	14
Pediatrics	12.7	9-10	11.5	10.9	14	13.4	9.4	13.5

Pain Mgmt: pain management; CLI: Coleman-Liau; NDC: New Dale-Chall; FKGL: Flesch Kincaid; FCS: FORCAST; G-FOG: Gunning FOG; NFC: New Fog Count; SMOG: Simple Measure of Gobbledygook. All articles were accessed June 2021.

**Table 3:** Readability assessment scores of patient education materials from the American Society of Regional Anesthesia and Pain Medicine, American Society of Anesthesiologists, Canadian Anesthesiologists' Society, and Society of Cardiovascular Anesthesiologists.

Category	CLI	NDC	FKGL	FCS	Fry	G-FOG	NFC	SMOG
ASRA	12.7	11-12	12.6	11	15	14.9	11.1	14.6
ASA	13	11-12	12.3	11.3	16	13.4	8.8	14.2
CAS	12.8	16+	15.5	11	16	15.9	13.3	16.4
SCA	12.7	13-15	15.4	11.1	15	17.9	16.1	16.4

CLI: Coleman-Liau; NDC: New Dale-Chall; FKGL: Flesch Kincaid; FCS: FORCAST; G-FOG: Gunning FOG; NFC: New Fog Count; SMOG: Simple Measure of Gobbledygook. All articles were accessed June 2021.

## Data Availability

The data used to support the findings of this study are available from the corresponding author upon request.
